# Targeting MALAT1 and miRNA-181a-5p for the intervention of acute lung injury/acute respiratory distress syndrome

This article has been retracted.

**DOI:** 10.1186/s12931-020-01578-8

**Published:** 2021-01-06

**Authors:** Yaling Liu, Xiaodong Wang, Peiying Li, Yanhua Zhao, Liqun Yang, Weifeng Yu, Hong Xie

**Affiliations:** 1 Department of Anesthesiology, The Second Affiliated Hospital of Soochow University, 1055 Sanxiang Road, Suzhou, 215004 Jiangsu China; 2 Department of Anesthesiology, Renji Hospital, Shanghai Jiaotong University School of Medicine, 160 Pujian Road, Shanghai, 200127 China; 3 Department of Cardiology, Shanghai East Hospital, Tongji University School of Medicine, Shanghai, China

**Keywords:** Acute lung injury, Lipopolysaccharide, Metastasis-associated lung adenocarcinoma transcript-1, miRNA-181a-5p, Factor associated suicide, Pro-inflammatory factor

## Abstract

**Background:**

ALI/ARDS is a severe lung injury leading to refractory respiratory failure, accounting for high morbidity and mortality. However, therapeutic approaches are rather limited. Targeting long non-coding RNA MALAT1 and microRNA miR-181a-5p might be potential option for ALI/ARDS intervention.

**Objective:**

We aimed to investigate the role of MALAT and miR-181a-5p in the pathogenesis of ALI/ARDS, and test the therapeutic effects of targeting MALAT and miR-181a-5p for ALI/ARDS intervention in vitro.

**Methods:**

MALAT1 and miR-181a-5p levels were measured in plasma from ALI/ARDS patients. In vitro human pulmonary microvascular endothelial cell (HPMEC) injury was induced by LPS treatment, and molecular targets of MALAT1 and miR-181a-5p were explored by molecular biology approaches, mainly focusing on cell apoptosis and vascular inflammation. Interaction between MALAT1 and miR-181a-5p was also detected. Finally, the effects of targeting MALAT1 and miR-181a-5p for ALI/ARDS intervention were validated in a rat ALI/ARDS model.

**Results:**

MALAT1 upregulation and miR-181a-5p downregulation were observed in ALI/ARDS patients. Transfection of mimic miR-181a-5p into HPMECs revealed decreased Fas and apoptosis, along with reduced inflammatory factors. Fas was proved to be a direct target of miR-181a-5p. Similar effects were also present upon MALAT1 knockdown. As for the interaction between MALAT1 and miR-181a-5p, MALAT1 knockdown increased miR-181a-5p expression. Knocking down of MALAT1 and miR-181a-5p could both improve the outcome in ALI/ARDS rats.

**Conclusion:**

MALAT1 antagonism or miR-181a-5p could both be potential therapeutic strategies for ALI/ARDS. Mechanistically, miR-181a-5p directly inhibits Fas and apoptosis, along with reduced inflammation. MALAT1 negatively regulates miR-181a-5p.

## Background

Acute lung injury (ALI)/acute respiratory distress syndrome (ARDS) is recognized as a severe respiratory syndrome associated with high morbidity and mortality due to heterogeneous pathologic factors [1]. Globally, ALI/ARDS affects approximately 3 million patients annually, accounting for 10% of intensive care unit (ICU) admissions and 23% of patients receiving mechanical ventilation in the ICU [2]. Pathologically, ALI/ARDS is characterized by a sustained excessive inflammatory process in the lung with increased alveolar capillary permeability, leading to pulmonary edema, hypoxemia, apoptosis and lung destruction [3, 4]. Unfortunately, treatment approaches are quite limited by far.

Non-coding RNA, including microRNA (miRNA) and long non-coding RNA (lncRNAs), is an increasing hot topic in lung inflammation and injury [5]. Initially identified as a marker of early metastasis in non-small-cell lung cancer [6], lncRNA metastasis-associated lung adenocarcinoma transcript-1 (MALAT1) is then found to regulate multiple process across multiple organs [7–9]. For example in the lung, MALAT1 participates in hyperglycemia-induced inflammatory response and apoptosis [10, 11], pneumonia [12], chronic obstructive pulmonary disease [13] and lung transplant-related ischemia–reperfusion injury [14]. Importantly, MALAT1 elevates in septic patients [15, 16] and preclinical septic mice [17]. Since the lung is a most vulnerable organ in septic injury, we hypothesize an important role of MALAT in ALI/ARDS pathogenesis.

A number of miRNAs have been implicated in the progression of lung disease [18]. MiRNA-181d was decreased in bronchial epithelial cells [19] from smokers, and miRNA-181a modulates inflammatory response in human fibroblasts [20, 21]. However, the role of miRNA-181 in ALI/ARDS and its interaction with lncRNA remain unclear, considering that lncRNA functions as competing endogenous RNAs (ceRNAs) or endogenous “sponge” RNAs in regulating the expression and biological functions of miRNAs.

A growing body of literature suggests that Fas signaling activation plays an important pathophysiological role in the development of inflammation and apoptosis in ALI/ARDS [22–25]. In the present study, we investigate the expression of MALAT1, miR-181a-5p, Fas and pro-inflammatory factors in ALI/ARDS patients, explored the molecular mechanism via which MALAT1 and miR-181a-5p participate in ALI/ARDS pathogenesis, and preliminarily evaluate the effects of targeting MALAT1 and miR-181a-5p in ALI/ARDS intervention.

## Materials and methods

### Synthesis of RNA nucleotides and plasmids

For MALAT1 knockdown, siRNA targeting MALAT1 (siR-MALAT1) and siR-NC (scramble) were designed and synthesized by GenePharma (Shanghai, China). For miR-181a-5p upregulation, mimic miR-181a-5p and mimic NC (miR30000256-4-5, miR40000256-4-5) were obtained from RiboBio (Guangzhou, China). Corresponding sequences are listed in Table 1.

**Table 1:** The sequence of primers

Name	Sequence
*Sequences of synthesized RNA nucleotides*	
siR-MALAT1-forward	5′-GGAGUACCCUGAAGCUAUAUU-3′
siR-MALAT1-reverse	5′-UAUAGCUUCAGGGUACUCCUU-3′
siR-NC-forward	5′-UUCUCCGAACGUGUCACGUUU-3′
siR-NC-reverse	5′-ACGUGACACGUUCGGAGAAUU-3′
mimic miR-181a-5p-forward	5′-AACAUUCAACGCUGUCGGUGAGU-3′
mimic miR-181a-5p-reverse	5′-UUUUGUAAGUUGCGACAGCCACU-3′
mimic NC-forward	5′-UUCUCCGAACGUGUCACGUTT-3′
mimic NC-reverse	5′-TTAAGAGGCUUGCACAGUGCA-3′
*Primers used in qRT-PCR*	
MALAT1-forward	5′-GCTCTGTGGTGTGGGATTGA-3′
MALAT1-reverse	5′-GTGGCAAAATGGCGGACTTT-3′
miR-181a-5p-forward	5′-ACACTCCAGCTGGGAACATTCAACGCTGTCGG-3'
miR-181a-5p-reverse	5′-TGGTGTCGTGGAGTCG-3′
Fas-forward	5′-CTGCATCATGATGGCCAATTCTGC-3′
Fas-reverse	5′-ATGACACTAAGTCAAGTTAAAGGC-3′
TNF-α-forward	5′-GCTGCACTTTGGAGTGATCG-3′
TNF-α-reverse	5′-TCACTCGGGGTTCGAGAAGA-3′
IL‐1β-forward	5′- CTGAGCTCGCCAGTGAAATG-3′
IL‐1β-reverse	5′-TGTCCATGGCCACAACAACT-3′
IL‐6-forward	5′-TTCTACAGACTACGGTTTGAG-3′
IL‐6-reverse	5′-GGATGACACAGTGATGCT-3′
U6-forward	5′-GCTTCGGCAGCACATATACTAAAAT-3′
U6-reverse	5′-CGCTTCACGAATTTGCGTGTCAT-3′
β-actin-forward	5′-AGAAAATCTGGCACCACACC-3′
β-actin-reverse	5′-CCATCTCTTGCTCGAAGTCC-3′

Previous studies have shown that lncRNAs function as ceRNAs or “sponges” to modulate miRNAs [26]. We used the Starbase V2.0 (http://starbase.sysu.edu.cn/) to predict that miR-181a-5p is the target RNA of MALAT1, and that Fas is the target gene of miR-181a-5p. Accordingly, the wide-type (WT) MALAT1 3′untranslated region (UTR) and its miR-181a-5p-binding-site mutant (MUT) were synthesized and cloned into the firefly luciferase-harboring pGL3 basic vector (Genomeditech, Shanghai, China) to create pGL3-MALAT1-WT and pGL3-MALAT1-MUT plasmids. Similarly, WT Fas 3′UTR and its miR-181a-5p-seeding-site MUT were synthesized and cloned into the same vector to create pGL3-Fas-WT and pGL3-Fas-MUT plasmids.

### In vivo and in vitro transfection

All siRNAs or mimic-RNAs or plasmids were dissolved by diethylpyrocarbonate-treated water to a final concentration of 40 μg/ml. A transfection mix was made of RNA nucleotides or plasmid with Lipofectamine 2000 (Invitrogen, Carlsbad, CA, USA) following manufacturer’s instructions. For in vivo transfection, the mix was injected intravenously 48 h prior to LPS treatment. For in vitro transfection, the mix was added to cell culture medium 24 h prior to LPS treatment.

### Human study

Human study was carried out in Shanghai East Hospital, Tongji University School of Medicine in China between March 1, 2016 and December 20, 2017, following the Ethical Principles for Medical Research Involving Human Subjects outlined in the Declaration of Helsinki. The ethics approval was obtained from the Ethics Committee of Shanghai East Hospital, Tongji University School of Medicine. Written informed consent was obtained from all participants. ALI/ARDS was diagnosed according to the Berlin Definition of ARDS [27].

The inclusion criteria were as follows: (1) ages > 18 and < 80 years old; (2) diagnosed as ALI/ARDS. Individuals were excluded if they (1) had pulmonary fibrosis; (2) had abnormal liver or renal function; (3) showed pneumonia according to the Clinical Pulmonary Infection Score (CPIS) [28]. The modified CPIS score is calculated from 5 variables (temperature, blood leukocytes, tracheal secretions, oxygenation and chest radiograph). A score of > 6 at baseline is suggestive of pneumonia; (4) had pulmonary edema due to cardiac dysfunction; and (5) needed extracorporeal membrane oxygenation (ECMO) support. For each patient, 2 ml of fresh blood was drawn into a vacuum tube containing ethylenediaminetetraacetic acid (EDTA) within 30 min after ALI/ARDS diagnosis. Whole blood samples were centrifuged at 3000×*g* for 15 min at 4 °C to precipitate blood cells. The plasma was then collected for further analyses. Healthy volunteers with comparable demographic parameters were enrolled as control group.

All ALI/ARDS patients received standard critical care, routine hemodynamic monitoring, and blood gas measurement. Mechanical ventilation (MV) was introduced when necessary. Demographic and clinical data were collected, including the patient’s gender, age, weight, pulse oxygen saturation (SPO_2_), duration of MV and the ratio of fraction of inspired oxygen to oxygen pressure (PaO_2_/FiO_2_). A bedside chest radiograph was taken every day.

### LPS-induced ALI in rats

This study was designed in accordance with ARRIVE guidelines. All rats received humane care, and procedures were approved by the Animal Care and Use Committee of the Tongji University School of Medicine. Male Sprague–Dawley (SD) rats (400–450 g) were housed at 22℃ to 24℃ of a 12:12 h light–dark circle, with at libitum access to food and water.

Rats were randomly assigned into seven groups: (1) sham, (2) lipopolysaccharide (LPS), (3) LPS + mimic NC, (4) LPS + mimic miR-181a-5p (5) LPS + siR-NC, (6) LPS + siR-MALAT1, and (7) LPS + mimic miR-181a-5p + siR-MALAT1 (n = 6 per group). 48 h after transfection, rats were anesthetized with 10% chloral hydrate (350 mg/kg, i.p.) and received i.p. injection of LPS (S1732-25, Beyotime, Shanghai, China) at 5 mg/kg or 0.9% saline solution. Arterial blood was obtained (0.3 ml) in heparinised syringes from the right femoral artery at 30 min before LPS treatment and 6 h and 12 h after LPS treatment for blood gas measurement. Rats were euthanized 12 h after LPS treatment and perfused the lungs were harvested and stored in liquid nitrogen for quantitative reverse transcription polymerase chain reaction (qRT-PCR) and Western blot measurements.

### Histopathological and immunohistochemical examination

The left superior lobes of the lung were fixed in 10% neutral buffered formalin for 24 h and embedded in paraffin. Tissues were cut into a series of microsections (4 μm), and then stained with haematoxylin and eosin (H&E) using standard protocols. The sections were then observed by a blinded pathologist under a light microscope (BXFM; Olympus, Tokyo, Japan) at a final magnification of 200x. The severity of lung injury was evaluated by a semi-quantitative histological index of quantitative assessment (IQA) of four grades ranging from 0–3, representing minimal, mild, moderate, and severe injury, respectively [29], in which the degree of alveolar edema, neutrophil infiltration and hyaline membrane formation were included.

Immunohistochemical staining for Fas was performed. In brief, sections from the right superior lobe of the lung were blocked with Peroxidazed® and incubated with Fas antibody (Beyotime, Shanghai, China) at 4℃ overnight. After washing with phosphate buffer solution (PBS, 2 × 5 min), slides were incubated with secondary antibody (10 min, Biocarta) and subsequently washed in PBS (2 × 5 min). Images were obtained with a light microscope (Olympus CH30, Olympus, Tokyo, Japan) at a final magnification of 200x. Immunoreactive density was analyzed with ImageJ software.

### Lung wet/dry weight ratio

The left lower lobe of the lung was excised and weighed to obtain the wet weight. Tissues were placed in an oven at 80 °C for 48 h until the weight became stable. The lobe was weighed again to obtain the dry weight, and the wet/dry ratio was calculated by the ratio of wet weight over the dry weight.

### Primary cell culture and drug treatment

Human pulmonary microvascular endothelial cells (HPMECs) were purchased from American Type Culture Collection (ATCC) and maintained in Dulbecco’s Modified Eagle’s medium (DMEM; Invitrogen, Carlsbad, CA, USA) containing 10% fetal bovine serum (FBS; Hyclone, Logan, UT, USA), 100 U/mL penicillin and 100 μg/mL streptomycin in a humidified atmosphere of 95% air and 5% CO_2_ at 37 °C. Cells were plated at 2.5 × 10^4^/cm^2^ prior to LPS treatment. LPS (50 ng/mL, S1732-25, Beyotime, Shanghai, China) was added to cells in glucose-free DMEM medium at 37℃ for 24 h.

### RNA extraction and qRT-PCR

The total RNA was isolated from the plasma of patients and volunteers, HPMECs and mouse lung tissues using TRIzol reagent (Invitrogen, Carlsbad, CA, USA). The RNA expression was measured immediately after extraction from patients or 12 h after LPS stimulation in rats and HPMECs. In brief, RNA was extracted using a small scale RNA extraction kit (Ambion, mirVana PARIS, USA) as previously reported [30]. RNA was then converted to first-strand cDNA using Mirvana miRNA Isolation Kit (Applied Biosystems, Foster City, USA). The cDNA was subjected to RT-PCR reactions wth the ABI7500 system (Applied Biosystems, Foster City, CA, USA) using the primers listed in Table. 1. The relative expression fold change of mRNAs was calculated by the 2^−ΔΔCt^ method normalized to U6 as internal control. Date were presented as expression level relative to control group.

### Western blot

Total protein was extracted from HPMECs using radioimmunoprecipitation assay (RIPA) analysis buffer, and qualified using a BCA protein assay kit (both from Beyotime, Shanghai, China). After denaturation, equal amount (20 μg/lane) of proteins were loaded and separated on 10% sodium dodecyl sulphate polyacrylamide gel electrophoresis. Proteins were then transferred to polyvinylidene difluoride membranes, blocked with 5% skim milk in a phosphate-buffered saline with Tween (PBST) solution (100 mM NaCl, 50 mM Tris, 0.1% Tween-20, PH 7.5) for 1 h at room temperature, and incubated with appropriate primary antibodies (anti-Fas, anti-tumor necrosis factor (TNF)-α, Santa Cruz, CA, USA; β-actin, Beyotime, China) overnight at 4℃. After wash, membranes were incubated with horseradish peroxidase (HRP) conjugated secondary antibodies (Sigma-Aldrich, Saint Louis, USA), and immunoreactive bands were visualised by enhanced chemiluminescence and analyzed with ImageJ software. The relative protein expressions were calculated after normalization with β-action. Data were presented as expression level relative to the control group.

### Measurement of HPMEC apoptosis

HPMECs were collected via trypsinization and stained with FITC-labelled anti-Annexin V and PI (both from BD Pharmingen, San Diego, CA, USA). After incubation at room temperature for 30 min in the dark, cells were immediately counted on a Flow Cytometer (Beckman Coulter, Inc., CA, USA). The dual dot plots were used to analyze the percentage of non-apoptotic cells (Annexin V−/PI−), early apoptotic cells (Annexin V + /PI−), late apoptotic cells (Annexin V + /PI +) and necrotic cells (Annexin V−/PI +).

### Luciferase reporter assay

pGL3-MALAT1-WT/MUT and pGL3-FAS-3′UTR-WT/MUT plasmids were co-transfected mimic miR-181a-5p/mimic NC in HMPECs. After 24 h, firefly luciferase activity was measured (Genomeditech, Shanghai, China). Data were presented as luciferase activity relative to the control group.

### Statistical analysis

Statistical analyses were performed using SPSS statistics, version 17.0 (IBM Inc., Chicago, IL) and GraphPad Prism 5.0 (GraphPad Software, Inc., San Diego, CA). The results were presented as mean ± SD if normal distribution or medians and interquartile ranges if non normal distribution for continuous variables, and as percentage for categorical variables. Continuous data were tested for normal distribution with the one-sample Kolmogorov–Smirnov test. One-way analysis of variance (ANOVA) was conducted in multiple group comparison. Fisher’s exact test was used to compare categorical data as appropriate. A Pearson correlation test was performed to determine the correlation between MALAT1 and miRNA-181a-5p. A P value < 0.05 was considered statistically significant.

## Results

### Increased MALAT1 and reduced miRNA-181a-5p expression in ALI/ARDS patients

Thirty ALI patients and fifteen healthy controls were recruited in the present study. Demographic characteristics of patients were comparable between ALI/ARDS group and the control group (Table 2). In ALI/ARDS patients, plasma MALAT1 level was significantly increased (Fig. 1a) and miR-181a-5p level was significantly decreased (Fig. 1b). Interestingly, the level of MALAT1 was inversely correlated with miRNA-181a-5p (Fig. 1c, Pearson’s correlation, R =  − 0.508, P = 0.0031), suggesting a possible interaction between them. We also detected the expression level of apoptotic receptor Fas and proinflammatory factors TNF-α, interleukin (IL)-1β and IL-6. As expected, we observed significant higher levels of them (Fig. 1d–g), consistent with the well-established ALI/ARDS associations of excessive tissue damage and inflammatory responses. Since ALI/ARDS is associated with vascular inflammation that contributes to diffuse alveolar damage in ALI/ARDS [31], we then moved on to explore the effects of miRNA-181a-5p on vascular injury in HPMECs, as well as the potential interaction between MALAT1 and miRNA-181a-5p.

**Table 2:** Clinical characteristics and biomarkers expression in ALI patients

Patient characteristics and pathological features	Total N 45	ALI		P value
		Yes 30	No 15	
Mean age ± SD (years)	57.2 ± 8.3	58.6 ± 8.5	57.1 ± 8.3	0.298
BMI (mean ± SD)	26.1 ± 2.4	26.3 ± 2.3	26.1 ± 2.4	0.719
Male	21 (46.6%)	15 (50.0%)	6 (40.0%)	0.391
Current smoker	30 (66.7%)	23 (76.3%)	7 (48.8%)	0.581
COPD	8 (17.7%)	6 (21.1%)	2 (10.6%)	0.058
Hypertension	13 (28.8%)	8 (28.9%)	5 (32.1%)	0.691
Chronic heart failure	5 (11.1%)	4 (13.2%)	1 (9.4%)	0.082
Diabetes	11 (24.4%)	8 (26.3%)	3 (23.3%)	0.689
Operation time: Mean ± SD (min)	182.1 ± 17.2	178.9 ± 13.6	N/A	N/A
Blood loss: Mean ± SD (ml)	280.2 ± 20.5	265.8 ± 21.4	N/A	N/A
ICU duration	7.2 ± 2.3	10.5 ± 2.6	N/A	N/A
Tracheal tube retaining time (days)	4.5 ± 1.6	5.8 ± 1.7	N/A	N/A
Relative MALAT1	1.8 ± 0.7	1.2 ± 0.7	2.5 ± 0.5	< 0.01
Relative miR-181a-5p	1.9 ± 0.2	2.3 ± 0.9	0.5 ± 0.1	< 0.01
Relative Fas	2.0 ± 0.4	1.3 ± 0.5	2.8 ± 1.2	< 0.01
Relative TNF-α	1.7 ± 0.5	2.9 ± 0.8	1.1 ± 0.3	< 0.01
Relative IL-1β	1.8 ± 0.6	2.2 ± 1.3	1.3 ± 0.8	< 0.01
Relative IL-6	1.6 ± 0.2	2.9 ± 0.5	1.7 ± 0.6	< 0.01

Continuous data are presented as mean ± SD, and numerical data are presented as numbers (percentage among total patients). P values were derived using a 2-sample Student’s t-test or Wilcoxon rank-sum test for continuous variables and 2-tailed χ^2^ or Fisher’s exact test for categorical variables. *Fas* factor associated suicide, *BMI* body mass index, *COPD* chronic obstructive pulmonary disease, *IL* interleukin, *MALAT1* metastasis-associated lung adenocarcinoma transcript-1, *TNF-α* tumour necrosis factor-α

**Fig. 1:** Increased expression of MALAT1 and decreased miRNA-181a-5p in ALI/ARDS patients. The RNA from plasma samples of patients was extracted and measured by qRT-PCR. (A-B) Increased MALAT1 expression and decreased miR-181a-5p expression in ALI/ARDS patients. (C) The negative correlation between MALAT1 and miRNA-181a-5p in ALI/ARDS patients determine by Pearson’s correlation (R =  − 0.508, P = 0.0031). (D-F) Increased expression of apoptotic receptor Fas and proinflammatory factors TNF-α, IL-1β and IL-6 measured by qRT-PCR in ALI/ARDS patients. *, ** p < 0.05, 0.01 vs control

### miR-181a-5p prevents LPS-induced apoptosis in HPMECs through directly targeting Fas

Previous studies have proved that miR-181a-5p could alleviate fibroblastic inflammation in non-ALI/ARDS models [20, 21]. We then hypothesized that miR-181a-5p exhibited similar protection focusing on endothelial apoptosis and apoptotic receptor Fas. To this end, HPMECs were cultured and subjected to LPS-induced injury to mimic ALI/ARDS. Mimic miR-181a-5p was transfected prior to LPS treatment. Mimic miR-181a-5p transfection resulted in upregulation of miR-181a-5p expression in HPMECs (Fig. 2a), confirming a successful transfection. As expected, this was brought down by LPS treatment, in concert with a decreased miR-181a-5p in ALI/ARDS patients (Fig. 1b).

**Fig. 2:** miRNA-181a-5p inhibits LPS-induced HPMEC apoptosis through directly targeting Fas. Mimic miR-181a-5p or mimic miR-NC was transfected to HPMECs, which were then treated with LPS. **a** Increased miR-181a-5p expression by mimic miR-181a-5p. **b** Decreased LPS-induced Fas mRNA level by mimic miR-181a-5p. **c** Decreased LPS-induced Fas protein level by mimic miR-181a-5p. **d** Decreased LPS-induced HPMEC apoptosis by mimic-miR-181a-5p. **e** pGL3-FAS-WT or pGL3-FAS-MUT plasmids were co-transfected with mimic miR-181a-5p or miR-NC. **f** Luciferase assay revealed that mimic miR-181a-5p decreased the luciferase activity in pGL3-FAS-WT but not in pGL3-FAS-MUT. *, **p < 0.05, 0.01.

Upon detection of Fas expression, we found that LPS increased Fas expression at both mRNA and protein levels, which were partially reversed by mimic miR-181a-5p transfection (Fig. 2b–d). Consistently, mimic miR-181a-5p also partially reversed LPS-induced apoptosis (Fig. 2e). These findings led us to further explore the molecular mechanisms via which miR-181a-5p prevented LPS-mediated cell death. With the help of Starbase V2.0, we predicted that Fas might be a direct target of miR-181a-5p. To test this, luciferase-harboring pGL3-FAS-WT or pGL3-FAS-MUT plasmids were co-transfected with mimic miR-181a-5p into HPMECs, and luciferase activity was detected. Interestingly, mimic miR-181a-5p could inhibit WT-Fas expression with no effects on MUT-Fas (Fig. 2r). Taken together, we proved that miR-181a-5p protects HPMECs against LPS-induced apoptosis though directly targeting and inhibiting Fas expression.

### miR-181a-5p prevents LPS-induced inflammation in HPMECs

We then explored the effect of miR-181a-5p on LPS-induced inflammation in HPMECs. Mimic miR-181a-5p was transfected prior to LPS treatment. We found that LPS induced significant increase in TNF-α expression at both mRNA and protein levels, which were partially reversed by mimic miR-181a-5p (Fig. 3a, b). Similar effects were also present in IL-1β and IL-6 mRNA levels (Fig. 3c, d), suggesting that miR-181a-5p protects HPMECs against LPS-induced vascular inflammation.

**Fig. 3:** miRNA-181a-5p alleviates LPS-induced inflammation in HPMECs. Mimic miR-181a-5p or mimic miR-NC was transfected to HPMECs, which were then treated with LPS. **a** Decreased LPS-induced TNF-α mRNA level by mimic miR-181a-5p. **b**, **c** Decreased LPS-induced TNF-α protein level by mimic miR-181a-5p. **d** Decreased LPS-induced IL-1β mRNA level by mimic miR-181a-5p. **e** Decreased LPS-induced IL-6 mRNA level by mimic miR-181a-5p. *, **p < 0.05, 0.01.

Taken together, we have proved that miR-181a-5p inhibits LPS-induced vascular inflammation and apoptosis, in which miR-181a-5p directly targets and inhibits Fas expression. We then move forward to explore the effects of MALAT1 on the above miR-181a-5p-targeting events.

### Knockdown of MALAT1 inhibits LPS-induced apoptosis in HPMECs

To explore the role MALAT1 on HPMEC apoptosis, cellular MALAT1 was knocked down by siR-MALAT1 transfection prior to LPS treatment. As expected, LPS increased MALAT1 expression, which was significantly downregulated by siR-MALAT1 (Fig. 4a), confirming a successful knockdown. Moving on to Fas and apoptotic analysis, LPS-induced FAS was inhibited by siR-MALAT1 at both mRNA level and protein level (Fig. 4b–d). Moreover LPS-induced apoptosis was also inhibited by siR-MALAT1 (Fig. 4e). These findings suggest a critical role of MALAT1 in LPS-mediated Fas upregulation and subsequent apoptosis.

**Fig. 4:** Knockdown of MALAT1 inhibits LPS-induced apoptosis in HPMECs. SiR-MALAT1 or siR-NC was transfected to HPMECs, which were then treated with LPS. **a** Decreased MALAT1 expression by siR-MALAT1. **b** Decreased LPS-induced Fas mRNA level by siR-MALAT1. **c**, **d** Decreased LPS-induced Fas protein level by mimic siR-MALAT1. **e** Decreased LPS-induced HPMEC apoptosis by siR-MALAT1. *, **p < 0.05, 0.01

### Knockdown of MALAT1 inhibits LPS-induced inflammation in HPMECs

We then explored the effect of MALAT1 on LPS-induced inflammation in HPMECs by knocking down of cellular MALAT1 with siR-MALAT1. We found that LPS-induced increase in TNF-α expression was inhibited by siR-MALAT1 at both mRNA level and protein level (Fig. 5a,b). Similar effects were also present in IL-1β and IL-6 mRNA levels (Fig. 5c,d), suggesting a critical role of MALAT1 in LPS-mediated vascular inflammation.

**Fig. 5:** Knockdown of MALAT1 inhibits LPS-induced inflammation in HPMECs. SiR-MALAT1 or siR-NC was transfected to HPMECs, which were then treated with LPS. **a** Decreased LPS-induced TNF-α mRNA level by siR-MALAT1. **b**, **c** Decreased LPS-induced TNF-α protein level by siR-MALAT1. **d** Decreased LPS-induced IL-1β mRNA level by siR-MALAT1. **e** Decreased LPS-induced IL-6 mRNA level by siR-MALAT1. *, **p < 0.05, 0.01

By far we have proved the critical role of MALAT1 on miR-181a-5p-targeting events, including apoptosis and vascular inflammation. Since lncRNAs function as ceRNAs or “sponges” to modulate miRNAs [26], we hypothesized the presence of MALAT1 and miR-181a-5p interaction.

### Interaction between MALAT1 and miR-181a-5p

Si-MALAT1 was transfected to HMVECs to detect the effect MALAT1 on miR-181a-5p expression. As expected, si-MALAT1significantly increased the expression of miR-181a-5p (Fig. 6a), suggesting that MALAT1 inhibit miR-181a-5p expression. However, when mimic miR-181a-5p was transfected to HMVECs, there was no effect of miR-181a-5p on MALAT1 expression (Fig. 6b). Interestingly, WT-MALAT1 could inhibit miR-181a-5p expression with no effects of MUT-MALAT1 suggesting the unilateral inhibition of MALAT1 on miR-181a-5p (Fig. 6c).

**Fig. 6:** Interaction between MALAT1 and miR-181a-5p. **a** SiR-MALAT1 or siR-NC was transfected to HPMECs, which were then treated with LPS. SiR-MALAT1 decreased miR-181a-5p expression. **b** Mimic miR-181a-5p or mimic miR-NC was transfected to HPMECs, which were then treated with LPS. Mimic miR-181a-5p failed to alter MALAT1 expression. **c** pGL3-MALAT1-WT or pGL3-MALAT1-MUT plasmids were co-transfected with mimic miR-181a-5p or miR-NC. Luciferase assay revealed that mimic miR-181a-5p decreased the luciferase activity in pGL3-MALAT1-WT but not in pGL3-MALAT1-MUT. *, **p < 0.05, 0.01

### Both miR-181a-5p and anti-MALAT1 improved outcome in ALI/ARDS rats

To further valid the translational value of the above findings in vivo, rat ALI/ARDS models were established by LPS i.p. injection at a dose of 5 mg/kg. Rats were sacrificed 12 h after LPS injection. H&E staining of the lung showed increased septal thickness, intra-alveolar transudates, and increased inflammatory cell infiltration (Fig. 7a, b). LPS group also exhibited increased Fas and TNF-α expression (Fig. 7c, d), suggesting increased apoptosis and inflammatory response in rat ALI/ARDS.

**Fig. 7:** miR-181a-5p and anti-MALAT1 improved outcome in ALI/ARDS rats. LPS was injected i.p. to induced ALI/ARDS in rats 48 h after transfection of mimic miR-181a-5p or mimic NC and siR-MALAT1 or siR-NC. **a**, **b** H&E staining showing increased septal thickness, intra-alveolar transudates, and increased inflammatory cell infiltration in LPS group. **c**, **d** Increased Fas and TNF-α protein expression in lung tissue extracts determined by Western blotting. **e** H&E staining showed that both miR-181a-5p and siR-MALAT1 improved LPS-induced lung injury. **f** IQA scores were reduced by both miR-181a-5p and siR-MALAT1. *, **p < 0.05, 0.01.

We then move on detect the effect of mimic miR-181a-5p and siR-MALAT1 on the outcome of rat ALI/ARDS. Rats were assigned into seven groups: (1) sham, (2) LPS, (3) LPS + mimic NC, (4) LPS + mimic miR-181a-5p (5) LPS + siR-NC, (6) LPS + siR-MALAT1, and (7) LPS + mimic miR-181a-5p + siR-MALAT1. As shown in Table 3, both mimic miR-181a-5p and siR-MALAT1 attenuated hypoxemia and hypercapnia of arterial blood gas, and reduced lung edema determined by wet/dry ratio. Lung histology showed that LPS induced destruction of alveolar wall and neutrophil infiltration, which were attenuated by both mimic miR-181a-5p and siR-MALAT1 (Fig. 7e), suggesting milder tissue destruction and alleviated inflammatory response. The IQA of seven groups were 0, 3 ± 1.1, 3 ± 1.8, 2 ± 0.9, 3 ± 1.5, 2 ± 0.8 and 1 ± 0.6 (group 4 vs. group 3, P < 0.05; group 6 vs. group 5, P < 0.05; group 7 vs. group 4, P < 0.05; group 7 vs. group 6, P < 0.05).

**Table 3:** Arterial blood gases (mmHg) and W/D in rats

Parameters	Sham	LPS	LPS + siR-NC	LPS + siR-MALAT1	LPS + mimic NC	LPS + mimic miR-181a-5p	LPS + siR-MALAT1 + mimic miR 181a-5p
PaO_2_							
30 min before LPS	125.8 ± 6.6	131.9 ± 7.2	135.8 ± 8.7	129.3 ± 3.2	133.2 ± 8.4	129.5 ± 6.1	130.4 ± 6.9
6 h after LPS	140.2 ± 7.9	84.8 ± 6.3*	99.6 ± 4.5*	114.8 ± 9.2*	80.4 ± 2.8*	119.5 ± 7.7*	135.4 ± 5.2
12 h after LPS	138.3 ± 5.5	68.2 ± 4.1**	75.6 ± 2.9**	89.6 ± 5.7**	74.7 ± 7.1**	97.5 ± 9.3**	126.6 ± 4.7
PaCO_2_							
30 min before LPS	33.1 ± 3.4	32.1 ± 3.1	38.6 ± 2.1	30.4 ± 5.6	37.4 ± 6.6	33.5 ± 8.1	34.6 ± 5.5
6 h after LPS	39.5 ± 2.0	50.3 ± 3.5*	53.3 ± 1.6*	42.4 ± 3.5	46.8 ± 4.8*	36.2 ± 2.2	35.4 ± 2.9
12 h after LPS	40.0 ± 3.2	55.1 ± 1.8*	57.8 ± 2.9*	42.5 ± 4.3	58.5 ± 6.2*	41.3 ± 4.5	40.9 ± 7.7
W/D	4.17 ± 0.94	6.25 ± 2.83*	6.56 ± 1.74*	5.14 ± 1.85*	6.72 ± 1.42*	4.98 ± 3.19	4.26 ± 3.24

Data are presented as mean ± SD. P values were calculated using analysis of variance on repeated measures. *LPS* lipopolysaccharide, *MALAT1* metastasis-associated lung adenocarcinoma transcript-1, *W/D* wet/dry ratio. *, **P < 0.05, 0.01 compared to sham group

For the immunohistochemical measurement, Fas expression was not evident in sham rats. Expression of Fas in the lungs was significantly higher in LPS, LPS + mimic NC and LPS + siR-NC rats than in LPS + mimic miR-181a-5p and LPS + siR-MALAT1 rats (group 4 vs. group 3, P < 0.05; group 6 vs. group 5, P < 0.05). Mimic miR-181a-5p plus siR-MALAT1 decreased Fas expression significantly compared to mimic miR-181a-5p or siR-MALAT1 alone (group 7 vs. group 4, P < 0.01; group 7 vs. group 6, P < 0.01) (Figs. 8, Fig. 9).

**Fig. 8:** miR-181a-5p and anti-MALAT1 decreased Fas expression in ALI/ARDS rats. LPS was injected i.p. to induced ALI/ARDS in rats 48 h after transfection of mimic miR-181a-5p or mimic NC and siR-MALAT1 or siR-NC. Lung immunohistochemical staining of Fas and its quantification revealed decreased Fas expression by both miR-181a-5p and siR-MALAT1.

**Fig. 9:** Immunoreactive density was analyzed with ImageJ software *, **p < 0.05, 0.01

Taken together, we confirm the translational value of antagonism of MALAT1 or promotion of miRNA-181a-5p, which could elicit therapeutic effects with a more favorable clinical outcome.

## Discussion

The present study demonstrated that lncRNA MALAT1 expression increased in ALI patients and LPS-induced rats and HPMECs, downregulating target miR-181a-5p, which, in turn, upregulated target gene Fas, promoting endothelial cell apoptosis, accompanying pro-inflammatory factors released.

Injury in pulmonary endothelial cells is critical component in diffuse alveolar damage (DAD), the hallmark pathology underlying ALI/ARDS [32]. Normal endothelial cells are highly selective with limited permeability, participating in forming the gas-blood barrier. In ALI/ARDS, DAD leads to the release of proinflammatory cytokines, which further recruit neutrophils to the lungs, exacerbating local and systemic inflammation and tissue injury [33]. Locally damaged endothelial cells allow for protein-rich fluid leaking into the alveoli and the interstitium, contributing to the devastating ALI/ARDS pathology [34]. In the present study, decreased miR-181a-5p and increased MALAT1 were detected in both ALI/ARDS patient plasma, leading us to further explore the HPMECs regarding these two RNAs. A logic gap of the current study is that, although miR-181a-5p and MALAT1 might be released by the endothelial cells to the plasma, we have no direct evidence proving the specific contribution of endothelial cells to plasma concentrations of miR-181a-5p and MALAT1.

Epigenetic factors play important roles in the development of hypoxia [7] and apoptosis [35, 36] which may contribute to ALI/ARDS pathogenesis. MicroRNAs are a kind of non-coding RNA with 22 to 29 bases involved in early development, cell proliferation, differentiation, apoptosis, energy metabolism and immune regulation [37]. MiRNA-181a-5p belongs to the miRNA-181 family, which has highly conserved gene sequence [38]. Decreased miR-181a-5p in both ALI/ARDS patient plasma and HPMECs after LPS stimulation suggests its role in ALI/ARDS pathogenesis. Importantly, we are the first to report that miR-181a-5p could directly target Fas and lead to subsequent apoptosis. Nevertheless, a kinetic delay may be present when measuring apoptosis in HPMECs, and one should be cautious when interpretating the data, as it might represent only the early phase apoptosis. This is another weak point of the present study. We also proved the role of miR-181a-5p in LPS-induced inflammatory response, which was in accordance with other studies. For example, in a pulmonary arterial hypertension rat model, miR-181a-5p expression was reduced and its upregulation significantly attenuated right ventricular remodelling and lung injury [39]. Another study found that both miR-181a-5p and miR-181a-3p were decreased in the atherosclerosis-induced vascular inflammation [40]. Furthermore, miR-181a-5p and miR-181a-3p cooperatively receded endothelium inflammation compared with single miRNA strand [40]. Taken together, miR-181a-5p demonstrated direct protection against ALI/ARDS via mitigating apoptosis and inflammation.

Recently, MALAT1 has been reported to participate in ALI/ARDS pathophysiology process. Inhibition of MALAT1 results in the suppression of inflammatory responses by upregulating miR-146a in LPS-induced ALI [41]. It also sponges miR-149 to promote inflammatory responses in LPS-induced ALI by targeting MyD88 [42]. These studies demonstrated the pivotal epigenetic role of MALAT1 in ALI/ARDS process.

One of the central concepts in ALI is that an unbalanced quantity or quality of the inflammatory response aggravates epithelial injury. In our results, the expression of MALAT1 was consistent with the TNF-α, IL-1β and IL-6, consistent with previous report [43]. IL-6 is a pro-inflammatory mediator that has been well discussed [44]. A vicious cycle between of MALAT1 and inflammatory was reported in other tissues. For example in cardiomyocytes, IL-6 induces MALAT1 overexpression in HL-1 cell response to LPS [45], and MALAT1 can enhance TNF-α expression at least partly via serum amyloid A-3 (SAA3) in LPS-treated cardiomyocytes [45].

MiR-181a-5p is the target miRNA of MALAT1 verified in myeloma cells [46]. In general, lncRNAs act as “molecular sponges” that compete with mRNAs for the binding of miRNAs and thus dampen the mRNA-destabilising potential of miRNAs. Although in the present study, the luciferase assay in plasmids confirm that miR-181a-5p, as a target of MALAT1, directly repressed Fas expression, there is little evidence to support the influence of miRNAs on lncRNAs.

An important contribution of the present article is that we performed a pilot study in vivo to test the translational value of the above findings in ALI/ARDS rats. Excitingly, down-regulation of MALAT1 or up-regulation of miRNA-181a-5p could inhibit apoptosis and inflammation, providing a more favorable clinical outcome. Similarly, MALAT1 deteriorates ARDS by upregulating intercellular adhesion molecule-1 (ICAM-1) expression via miR-150-5p downregulation [47]. These results were in accordance with studies on other organs. In a study of hepatic ischemia–reperfusion injury, increased inflammatory reaction triggered by hypoxia/reoxygenation stimulation was also abrogated following MALAT1 suppression associated with mitigated inflammatory response [48]. MALAT1 targets TLR4 which regulates the inflammation and cell apoptosis of rat pulmonary microvascular endothelial cells via nuclear factor (NF)-κB and p38 mitogen activated protein kinase (MAPK) signaling pathway [49].

Limitations of the present study includes lack of cell type specificity for MALAT1 and miR-181a-5p. In addition, we did not assess long-term ALI/ARDS prognosis in both humans and rats. Future studies could try to pinpoint the specific cell type for MALAT1 target, and evaluate if targeting MALAT1 and miR-181a-5p provide long-term protection with decreased complications such as pulmonary fibrosis.

## Conclusions

The present study demonstrates that downregulation of MALAT1 and upregulation of miR-181a-5p could both be potential therapeutic strategies for ALI/ARDS. Mechanistically, miR-181a-5p directly inhibits Fas and apoptosis, along with reduced inflammation. MALAT1 negatively regulates miR-181a-5p. We can foresee real-time clinical interventions performed at the time of ALI that take advantage of antagonism of MALAT1.

## Data Availability

The data is available on the request.

## Abbreviations

ALI: Acute lung injury
ANOVA: One-way analysis of variance
ARDS: Acute respiratory distress syndrome
ATCC: American type culture collection
ceRNAs: Competing endogenous RNAs
CPIS: Clinical pulmonary infection score
DMEM: Dulbecco’s modified eagle’s medium
ECMO: Extracorporeal membrane oxygenation
EDTA: Ethylenediaminetetraacetic acid
FBS: Fetal bovine serum
FiO_2_: Fraction of inspired oxygen
HPMECs: Human pulmonary microvascular endothelial cells
HRP: Horseradish peroxidase
H&E: Haematoxylin and eosin
ICAM-1: Intercellular adhesion molecule-1
ICU: Intensive care unit
IL: Interleukin
IQA: Index of quantitative assessment
lncRNA: Long non-coding RNA
LPS: Lipopolysaccharide
MALAT1: Metastasis-associated lung adenocarcinoma transcript-1
MAPK: Mitogen activated protein kinase
miRNA: MicroRNA
MUT: Mutant
MV: Mechanical ventilation
NF-κB: Nuclear factor-κB
PaO_2_: Oxygen pressure
PBST: Phosphate-buffered saline with tween
qRT-PCR: Quantitative reverse transcription polymerase chain reaction
RIPA: Radioimmunoprecipitation assay
SAA3: Serum amyloid A-3
SD: Sprague–Dawley
SPO_2_: Pulse oxygen saturation
TNF-α: Tumor necrosis factor-α
UTR: Untranslated region
WT: Wide-type
